The article "Dysregulation of lncRNA in Helicobacter pylori-Infected Gastric Cancer Cells" was published in 2021. Journal: Biomed Res Int.

# Dysregulation of lncRNA in *Helicobacter pylori*-Infected Gastric Cancer Cells

**DOI:** 10.1155/2021/6911734

**Published:** 2021-07-09

**Authors:** Leila Yousefi, Hamid Owaysee Osquee, Reza Ghotaslou, Mohammad Ahangarzadeh Rezaee, Tahereh Pirzadeh, Javid Sadeghi, Fatemeh Hemmati, Bahman Yousefi, Seyyed Yaghoub Moaddab, Mehdi Yousefi, Masoud Shirmohammadi, Mohammad Hossein Somi, Khudaverdi Ganbarov, Hossein Samadi Kafil

**Affiliations:** ^1^Student Research Committee, Faculty of Medicine, Tabriz University of Medical Sciences, Tabriz, Iran; ^2^Pharmaceutical Nanotechnology Research Center, Faculty of Medicine, Tabriz University of Medical Sciences, Tabriz, Iran; ^3^Immunology Research Center, Faculty of Medicine, Tabriz University of Medical Sciences, Tabriz, Iran; ^4^Stem Cell Research Center, Faculty of Medicine, Tabriz University of Medical Sciences, Tabriz, Iran; ^5^Liver and Gastrointestinal Diseases Research Center, Faculty of Medicine, Tabriz University of Medical Sciences, Tabriz, Iran; ^6^Department of Microbiology, Baku State University, Baku, Azerbaijan; ^7^Drug Applied Research Center, Faculty of Medicine, Tabriz University of Medical Sciences, Tabriz, Iran

## Abstract

*Helicobacter pylori* (*H. pylori*) infection is the most common cause of gastric cancer (GC). This microorganism is genetically diverse; GC is caused by several genetic deregulations in addition to environmental factors and bacterial virulence factors. lncRNAs (long noncoding RNAs) are significant biological macromolecules in GC, have specific functions in diseases, and could be therapeutic targets. Altered lncRNAs can lead to the abnormal expression of adjacent protein-coding genes, which may be important in cancer development. Their mechanisms have not been well understood, so we are going to investigate the risk of GC in a population with both high lncRNA and *H. pylori* infection.

## 1. Introduction

*Helicobacter pylori* (*H. pylori*) is a Gram-negative motile curved microorganism [1] that causes a variety of diseases such as cancer in the gastric mucosa, peptic ulcers, gastritis, and mucosa-associated lymphoid tissue lymphoma (MALT) [2, 3]. In spite of the close relationship between *H. pylori* infection and progression of gastric malignancies [4], the mechanisms of this process are not thoroughly clear.

GC is one of the most common cancers and death agents worldwide [3, 5–7]. In East Asia, including China, its prevalence is high [8]. In 2015, 498,000 new deaths in association with GC were reported in China [5]. *H. pylori* infection is the most common cause of GC [3, 5]. Some types of *H. pylori*, like vacuolating cytotoxin (VacA) and cytotoxin-associated gene- (cagA-) positive subtypes, are most associated [5]. The cag pathogenicity island (cag PAI), one of the most important virulence factors of *H. pylori*, has 31 significant genes, including two regions, cag-I and cag-II [9]. Between these two regions is located an insertion sequence (IS) element, IS605 transposases (tnpA and tnpB); its virulence levels are different [9]. In Iran, for the first time, Abadi et al. detected an association between *tnp*A and *cag*A genes with GC [10]. In Peruvian and Brazilian patients, among gastrointestinal diseases, GC had an uppermost frequency of the *tnp*A gene [11, 12]. Ghotaslou et al. revealed that the rate of *tnp*B in GC is high [9]. To the best of our knowledge, this is the first time that the high prevalence of the *tnp*B gene in GC patients is reported [9]. The cagA genotype has various prevalence, and in GC patients, it has been shown to be between 50 and 100% [9]. Also, the prevalence of *cag*A in Ghotaslou et al.'s study was 65.2%, and it was mostly found in *H. pylori* isolated from GC and chronic gastritis (CG) patients [9].

The article "Dysregulation of lncRNA in Helicobacter pylori-Infected Gastric Cancer Cells" was published in 2021. Journal: Biomed Res Int.

In two independent researches from Taiwan and Brazil, the prevalence of the *cag*A gene in GC has been reported to be 100% and 35%, respectively [11, 13]. The differences in virulence genes were probably related to geographical regions, patient number, polymerase chain reaction (PCR) conditions, primer sets, and strains [9].

*H. pylori* is genetically diverse [9]; GC is caused by several genetic deregulations in addition to environmental factors and bacterial virulence factors [14]. *H. pylori* excites an inflammatory response in the gastric mucosa and can affect gastric lesion [15]. Hypochlorhydria and gastric atrophy, two types of gastric precancerous lesions, are caused by *H. pylori* infection [16]. A low number of infected individuals develop cancer, indicating that genetics has an important role in the gastric pathogenesis [16, 17]. However, the pathogenesis of GC associated with *H. pylori* is not completely understood. In order to prevent, diagnose, and treat GC, we can help from molecular pathways. This review focuses on lncRNAs which are dysregulated in *H. pylori*-infected GC cells [15].

Gastric cancer (GC) is the fourth most common cancer and the second cause of cancer-related death [18]. About 95% of gastric tumors are adenocarcinomas [19]. Environmental factors have an important role in the carcinogenesis. Among the environmental factors, diet and infection with *H. pylori* are the most common suspects in gastric tumorigenesis [18]. Also, GC is a complex, multistep process involving dysregulation of oncogenic pathways. These oncogenic signaling pathways can be activated through genetic and epigenetic changes [20, 21]. Genetic changes, like gene mutations, gene amplification, deletions or allelic loss, and chromosomal translocations, can cause gain of function in oncogenes and loss of function in tumor suppressor genes, finally involved in gastric carcinogenesis [21, 22]. Gastric cancer involves the surface of epithelial cells in the stomach. Each site of the stomach can contain cancer, but the gastric antrum and pylorus show the highest incidence of gastric cancer. However, the occurrence of gastric cancer is a complex process of progressive development that includes multiple factors, multiple steps, and coding and noncoding genes [23].

The article "Dysregulation of lncRNA in Helicobacter pylori-Infected Gastric Cancer Cells" was published in 2021. Journal: Biomed Res Int.

## 2. Coding and Noncoding RNA

Most of the DNA in human cells is transcribed into RNA, but only about 2% is translated into protein and the rest of the RNA is called noncoding RNA (ncRNA) [3]. Many ncRNAs have been found and shown to act in gene regulation [24] and play important roles in cancer development [4]. This class of RNA species includes microRNA (miRNA) and lncRNAs [24]. The biological function of miRNA is well known, but lncRNAs are new issues that have not been well studied.

miRNAs have short length, are involved in posttranscriptional regulation, and affect significantly on multiple biological functions [25]. A lot of miRNAs participate in *H. pylori*-related gastric pathology by being involved in the expression of target messenger RNAs (mRNAs) [25].

It is estimated that about two-thirds of the genes and also approximately 60 percent of genes encoding human protein are manipulated by miRNAs. These miRNAs always target one mRNA or multiple mRNAs and degrade or inhibit the translation of mRNAs. Moreover, they control the expression of genes at the translation level. Previous studies show that the miRNA level in tissues, cells, and body fluids is a biomarker for early diagnosis, treatment, and prognosis of tumors [26, 27].

Recently, in a study, *H. pylori* infection-associated diseases based on the miRNA-mRNA interaction network were investigated. miRNA levels in *H. pylori*-infected patients with gastritis, duodenal ulcer, gastric cancer, or mucosa-associated lymphoid tissue lymphoma were measured. Thirty-four miRNAs were identified, and investigating those miRNA target genes showed that *H. pylori* infection was significantly associated with cancer and regulation of mRNA synthesis. The miRNA-mRNA interaction network was produced, and 765 miRNA target genes were obtained. Target genes including *BCL2*, *MYC*, *ZEB2*, *MALAT1*, *HMGA2*, *CCND2*, *CDKN1A*, *VEGFA*, *PTEN*, and *ZEB1* were the most connected with miRNAs in this network. These miRNAs and target genes may have significant roles during *H. pylori* infection [28].

The article "Dysregulation of lncRNA in Helicobacter pylori-Infected Gastric Cancer Cells" was published in 2021. Journal: Biomed Res Int.

Also, another various noncoding RNA has been discovered. Some of them are as follows: piwi-interacting RNA (piRNA), small nucleolar RNAs (snoRNA), transfer RNA (tRNA), small nuclear RNA (snRNA), transcribed ultraconserved noncoding RNAs (T-UCR), telomerase RNA (TERC), and ribosomal RNA (rRNA). Their transcript length is varied from 25 nt (piRNA) to 5070 nt (rRNA) [29, 30].

## 3. lncRNAs

lncRNAs generally are RNA macromolecules with their transcript length exceeding 200 nt and have no coding ability [3, 4, 31]. lncRNAs are significant biological macromolecules in GC [32], have specific functions in diseases, and could be therapeutic targets [24]; their mechanisms have not been well understood.

Recently, it has been shown that considerably expressed lncRNAs are related to various diseases, including infectious diseases, neurological disorders, inflammatory diseases, autoimmune diseases, cardiovascular diseases, and different cancers [25] (Figure 1). Altered lncRNAs can lead to the abnormal expression of adjacent protein-coding genes, which may be important in cancer development [33]. Since lncRNAs have an important role in the control of cellular processes, they are dysregulated in a variety of cancers [34]. The lncRNA growth arrest special 5 (GAS5), which in human cancers has a radical inhibitory role, has been reported to interfere in the carcinogenesis development of several cancers, such as prostate cancer, hepatocellular carcinoma, colorectal cancer, and breast cancer [34].

lncRNAs, according to genomic organization, can be divided into various subtypes such as intergenic lncRNAs, intragenic lncRNAs, and enhancer lncRNAs (elncRNAs) (Table 1) [35]. Long intergenic noncoding RNA (lincRNA), the main type of the lncRNA family, like LINC00152 is highly expressed in cancer tissues. Its transcript length is 828 nt [36]. lncRNAs can influence genes in the same chromosome or in other chromosomes (20). Some intergenic lncRNAs seem to control the expression of both near and remote genes [37].

These lncRNAs have been found to regulate the levels of genomically neighboring (*cis*-acting) or distal (*trans*-acting) gene products via a variety of molecular mechanisms that are either transcript-dependent or transcription-dependent. The function of a transcription-dependent lncRNA depends on the act of transcription alone and does not rely on transcript sequence [38].

Intragenic lncRNA like RUNX1 overlapping RNA (RUNXOR) attaches to promoters and enhancers of the runt-related transcription factor 1 (RUNX1) gene [39]. RUNXOR is regulated highly in AML samples. RUNXOR through the 3′-terminal fragment interacts directly with the RUNX1 promoter and enhancers and contributed in the orchestration of an intrachromosomal loop. The 3′ region of RUNXOR also has a role in long-range interchromosomal interactions with chromatin regions that are involved in multiple RUNX1 translocations. This information suggests that RUNXOR noncoding RNA may serve as a previously unidentified candidate component that participates in chromosomal translocation in hematopoietic malignancies [40].

elncRNAs are transcribed from enhancer regions and have high monomethylation of histone H3 lysine 4 (H3K4me1). The expression of elncRNAs is also related to the activation of the enhancers as determined by H3K27Ac. Importantly, developmental and signal-dependent changes in elncRNA expression are highly correlated with the expression of target genes, particularly in the heart. Therefore, elncRNAs are expressed upon developmental differentiation cues and upon signal transduction events organized by signal-dependent transcription factors or nuclear receptors. Also, elncRNAs could participate in the initiation and stabilization of the loop, which finally determines the integration of enhancers within gene regulatory networks. In contrast, many elncRNAs are not required for the looping process itself. Instead, elncRNAs act once the loop is already formed, in order to facilitate RNAPII pause release at target transcriptional start sites and to promote transcriptional elongation. However, the mechanisms suggest *cis*-regulatory function for elncRNAs. Indeed, the main characteristics of elncRNAs, including their low expression, their absence at genomic regions other than their site of transcription, and the minimal effects of loss of function on nonadjacent coding genes, are mainly consistent with a predominant *cis* mechanism of action. Therefore, elncRNAs could exert their function via promoting direct interactions between enhancers and neighboring or distal genomic regions, refined within specific three-dimensional domains [35, 41, 42].

The article "Dysregulation of lncRNA in Helicobacter pylori-Infected Gastric Cancer Cells" was published in 2021. Journal: Biomed Res Int.

Another subtype, antisense lncRNAs by DNA–RNA, RNA–RNA, or protein–RNA interactions, controls nearly every level of gene regulation. Also, antisense lncRNAs by different mechanisms contribute to the regulation of the expression of their close genes in *cis* or more distant genes in *trans*. Antisense lncRNAs contribute in various functions, like X-inactivation, imprinting, and epigenetic regulation.

Albeit most lncRNAs have similarities with mRNAs such as transcript processing, the 5′ cap structure and 3′ poly(A) tail have been newly identified lncRNAs that have different mechanisms, for example, some of them are capped by snoRNAs at both ends or form circular RNA structures. Some classes of lncRNAs, including enhancer RNAs (eRNAs) and circular intronic RNAs (ciRNAs), do not have poly(A) tail [42–44].

circRNAs have multiple notable characteristics, including diversity, encoding by different genes with different sizes and expression levels. The spliced circle molecule has varied sizes from under 100 nt to over 4 kb. One circRNA has been identified to be related to disease phenotype. ANRIL, a long noncoding RNA, encodes circular variants. The expression of circular ANRIL (cANRIL) is associated with atherosclerotic vascular disease risk.

ciRNAs are intron lariats that have been circularized. Some ciRNAs improve the transcription of the genes which they are derived [45].

## 4. Gene Imprinting

In most imprinted clusters, there is an lncRNA [46]. lncRNAs, including Airn, Kcnq1ot1, Ube3aas, Ipw, Zfp127as, PEC2, PEC3, Pwcr1, Nespas, Exon1A, miR-296, miR-298, and H19, are associated with imprinted gene clusters [46]. Some of the lncRNAs control imprinting through improving sectionalization of intrachromosomal higher-order chromatin, contributing in replication timing and subnuclear settling. But the mechanism of other lncRNAs is regulation by transcriptional occlusion. By this function, the lncRNAs participate in vital biological processes such as placental and embryonic growth, pluripotency maintenance, cell differentiation, and synaptic development and plasticity [47].

## 5. X-Inactivation

X-inactivation is one of epigenetic processes that causes disease when abnormally dysregulated [48]. One of the exemplary cases from lncRNA biological functions is X-inactivation. The mechanisms of this process are exertion of chromatin modifiers, formation of RNA-based subnuclear compartments, and control of transcription via antisense transcription. Furthermore, XCI and lncRNAs newly seem to be in relation to the development of cancer [49].

The lncRNA XIST (X-inactive-specific transcript) is a product of the XIST gene and the master regulator of X-inactivation in mammals [50, 51]. In a survey, the relationship between lncRNA XIST expression and clinicopathological characteristics was investigated in gastric cancer patients and lncRNA XIST was markedly overexpressed in gastric cancer tissues [52].

## 6. Autophagy Regulation

Autophagy is a process that participates in maintaining homeostasis for environmental stresses like chemical and physical damage and nutrient shortage [53, 54]. Some lncRNAs are involved in this process. Up to now, over 37 autophagy-related (ATG) genes have been found in yeast and most of their orthologs exist in mammals. There is a relationship between lncRNAs and ATG genes in four steps of autophagy, including initiation, phagophore nucleation, autophagosome elongation/closure, and autolysosome fusion. Downregulation of *H19* enhances the expression of Beclin 1 (mammalian ortholog of ATG6) and ATG7 that can be a good marker for the next investigation of the relationship between *H19* and autophagy. An artificial long noncoding RNA (AlncRNA), Ad5-AlncRNA, has been identified that its high expression activates autophagy. IFN-*γ* released through *Mycobacterium bovis* bacillus Calmette-Guérin (BCG) can inhibit lncRNA maternally expressed gene 3 (MEG3), leading to the activation of autophagy and increasing eradication of intracellular *Mycobacterium bovis* BCG. Also, similarly in macrophages, tumor cells may induce autophagy in order to survive under different stresses via inhibiting *MEG3*. In fact, the level of *MEG3* expression is strikingly decreased in bladder cancer cells, as a result enhancing autophagy and cell proliferation. Moreover, *MEG3* also through repressing autophagy in human glioma cells promotes cisplatin-induced apoptosis [53].

The article "Dysregulation of lncRNA in Helicobacter pylori-Infected Gastric Cancer Cells" was published in 2021. Journal: Biomed Res Int.

ATGs, like LC3, Beclin 1, ATG5, and ATG7 that play important roles in autophagy, are abnormally expressed in GC and are used as signs of autophagy in this cancer. In GC cells, overexpression of ATG5 increases chemoresistance [55].

## 7. lncRNAs in *H. pylori*-Infected GC Cells

Up-to-date diagnosis and treatment of GC have been a critical issue, so it is better to understand well the effect of expression levels of lncRNA in GC cells. In this review, we are going to investigate the risk of GC in a population with both dysregulated lncRNA and *H. pylori* infection.

A study that for the first time investigated linked influence between expression levels of lncRNA in serum and *H. pylori* infection on risk of GC found that there is an association between high expression of H19 and LINC00152 levels and risk of GC, and also, the risk of GC in a population with both high lncRNA and *H. pylori* infection is increased [5]. In 2016, H19 and LINC00152 levels were evaluated in a Chinese population with *H. pylori*-associated gastric cancer and it has been shown that lncRNA is a significant cancer biomarker [5].

Some recent researches reported that inapt expression of some lncRNAs like survival-associated mitochondrial melanoma-specific oncogenic RNA (SAMMSON), HOX transcript antisense intergenic RNA (HOTAIR), and gastric adenocarcinoma predictive long intergenic noncoding RNA (GAPLINC) may be a diagnostic biomarker for therapy of GC [3]. Recently, in China, a study determined that a kind of lncRNA, THAP9 antisense RNA 1 (THAP9-AS1), which is stimulated in *H. pylori* infection, has an important role in the proliferation of GC cells. Since THAP9-AS1 in GC tissue was higher than that in gastritis tissue, it shows that THAP9-AS1 has a functional role in the development of GC [3].

The article "Dysregulation of lncRNA in Helicobacter pylori-Infected Gastric Cancer Cells" was published in 2021. Journal: Biomed Res Int.

Circulating lncRNAs are expressed abnormally in GC patients. These lncRNAs seem to be promising biomarkers for early detection of GC [56]. Plasma H19 and *long intergenic non-protein-coding RNA152* (LINC00152) are the main circulating lncRNAs that are expressed highly in GC patients. H19 by binding to RUNX1 and Isthmin1 (ISM1) improves GC cell proliferation, migration, and invasion, showing that H19 functions as an oncogene in GC. Fer-1-like family member 4 (pseudogene) (FER1L4), cancer upregulated drug-resistant (CUDR) gene, long stress-induced noncoding transcript 5 (LSINCT-5), and phosphatase and tensin homolog pseudogene 1 (PTENP1) are the main downregulated circulating lncRNAs in GC [56]. The secretion mechanism of lncRNA has not been studied absolutely. Probably, they are secreted in a manner similar to miRNAs. Newly circulating lncRNAs have been found in exosomes that could be protected from RNase. In the secretion pathway, apoptotic bodies and microvesicles may also contribute. Circulating lncRNAs may serve as important signal-conducting molecules in several physiological and pathological processes [56].

In a study, the circulating expression level of HULC (highly upregulated in liver cancer) was investigated in the serum of GC patients and its clinical importance as a serum biomarker for diagnosis and prognosis of GC was found. Also, the level of HULC in serum was higher in *H. pylori*-infected patients [57].

lncRNA acts as a tumor inhibitor and oncogene in the progress of GC [5]. lncRNA by affecting DNA, RNA, and protein has an important role in cell proliferation, apoptosis, and immune response [2]. lncRNA by various mechanisms like chromatin remodeling, RNA processing, translation, mRNA stability, and interacting with proteins has a serious role in the progress of GC [3]. lncRNA is also involved in other biological functions such as genome packaging, genome rearrangement, gene imprinting, and dosage compensation [6]. The expression of lncRNA in *H. pylori*-infected GC shows that probably there are different pathogenesis mechanisms between *H. pylori*-positive and *H. pylori*-negative GC [58]. Carcinogenesis of GC is associated with multiple lncRNAs like HOTAIR, H19, PTENP1, and GAS5 [59]. LINC00673 could be a tumor inhibitor in GC, but the rs11655237 A allele inhibits the transcription of LINC00673 [59]. Zhu et al. found that XLOC_014388 and XLOC_004122, two differentially expressed lncRNAs, in *H. pylori*-infected tissues, probably contribute in the immune response against *H. pylori* infection [25].

The article "Dysregulation of lncRNA in Helicobacter pylori-Infected Gastric Cancer Cells" was published in 2021. Journal: Biomed Res Int.

Prostate cancer noncoding RNA 1 (PRNCR1), an lncRNA transcribed from 8q24, by activating the androgen receptor (AR), contributes in the carcinogenesis of prostate cancer, and polymorphisms in the lncRNA PRNCR1 are a risk for different cancers such as prostate cancer, colorectal cancer, and gastric cancer (8). Also, in the 8q24 region, lncRNAs prostate cancer-associated transcript 1 (PCAT1) and colon cancer-associated transcript 2 (CCAT2) by affecting DNA break repair and chromosome instability play a role in cancer development, and polymorphisms in these lncRNAs were crucial risks of cancers [8]. Based on this knowledge, in a study, the susceptibility of polymorphisms (PRNCR1: rs7463708, rs7007694, rs16901946, and rs13252298; PCAT1: rs1026411 and rs12543663; CCAT2: rs6983267) in the lncRNAs in the region of 8q24 was investigated to risk of gastric cancer [8]. The genotype of rs16901946 was crucially different, and the G allele carriers were related to higher risk of gastric cancer [8].

A lot of investigations have discovered that miRNA and posttranscriptional regulation of noncoding RNA contribute effectively in the development of cancer, which has become a research field related to the pathogenesis of GC including *H. pylori*-related GC [58]. Chu et al. in 2011 suggested the hypothesis of competing endogenous RNA (ceRNA) that became a hot subject in researches [58]. The ceRNA network is regulated during development of tumors, including ovarian cancer, colon cancer, and GC [58]. Since the regulation of noncoding RNA related to *H. pylori* in GC has not been thoroughly studied, ceRNA regulation in this case is largely unknown. Recently, in China, the ceRNA regulatory network of GC with and without *H. pylori* infection and also relevant genes has been explored by Chu et al. From 32 differentially expressed mRNAs (DEmiRNAs), the expression of 21 cases was decreased and 11 increased. There were 27 differentially expressed lncRNAs (DElncRNAs) (24 DElncRNAs downregulated and 3 upregulated) and 257 DEmRNAs screened out [58]. LINCO1254, LINCO1287, LINCO1524, and U95743.1 were expressed highly in GC patients with *H. pylori* rather than without *H. pylori* [58].

In a Chinese population, it has been shown that LINC00673 rs11655237 enhances the risk of GC [59], by producing a binding site for miR-1231 downregulating LINC00673 expression [59]. This shows that, in the GC process, there is a significant interaction between lncRNAs and miRNAs; also, a significant relationship between rs11655237 and *H. pylori* infection is a risk for GC [59].

Recently, a study showed that H19 is a critical regulatory molecule in tumorigenesis [4]. H19 overexpression in *H. pylori*-infected GC cells by increasing nuclear factor kappa B- (NF-*κ*B-) induced inflammation elevated proliferation and invasion of these cells and also decreased apoptosis [4, 24]. In spite of H19 not having an open reading frame, it contains a secondary RNA structure which is much in the human placenta and several fetal tissues and may have a fundamental role in embryogenesis, fetal growth, and tumor progress [24]. Studies have shown that the expression of H19 in some types of cancers like colon, bladder, and breast cancer is high. However, radical role and mechanism of H19 in GC are vague [24]. H19 contains usual and unusual binding sites for the let-7 family of microRNAs that has a significant role in cancer and metabolism. The expression of miR-141 is reduced in GC and increases in epithelial ovarian cancer, which is different in various tumors and cell types. In 2015, in China, the relation between H19 and miR-141 was investigated and it was found that H19 and miR-141 compete for binding to each other's targets, which had a crucial role in GC progression [24]. Knowing the correlation between miRNA and lncRNA would contribute to diagnosis and therapy of cancers based on miRNA/lncRNA [24].

The article "Dysregulation of lncRNA in Helicobacter pylori-Infected Gastric Cancer Cells" was published in 2021. Journal: Biomed Res Int.

In a study for analyzing lncRNA AF147447 expression in *H. pylori* infection, it was measured after *H. pylori* coculture with GC cells. Its expression was decreased in three gastric epithelial cells [60]. The AF147447 expression in *H. pylori*-positive gastric tissues was investigated in mice. During infection, the AF147447 expression was in its low level [60]; lncRNA AF147447 prevented cell proliferation and cell migration both in vitro and in vivo [60].

The binding of *H. pylori* to the host tissue is critical for colonization and causing disease [61]. *H. pylori* by binding to the gastric mucosa influences the gastric microenvironment [62]. The gastric epithelium is protected by mucins that are a kind of glycoproteins [61]. The gastric mucin includes apomucin and O-linked carbohydrate side chain [62]. Twelve genes encode apomucins. Several of them, MUC1, MUC5AC, and MUC6, are present in healthy gastric tissue, and MUC2 is concentrated in a part of healthy gastric tissue but is usually present in the duodenum [62]. Since *H. pylori* prevents the expression of MUC5AC and MUC1 genes, mucin in the surface of the stomach is lowered [61]. In *H. pylori*-infected MKN45 cells, the expression of MUC2 is increased [63]. So the variations in mucin expression could be prognostic markers of gastric cancer. Some of MUC2 are present in the gastric antrum [62]. Those surveys suggested that *H. pylori* through MUC5AC colonizes the stomach, and MUC5AC is a part of the defense system in the gastric mucosa [62, 64].

The article "Dysregulation of lncRNA in Helicobacter pylori-Infected Gastric Cancer Cells" was published in 2021. Journal: Biomed Res Int.

In investigating the ability of lncRNA AF147447 for altering miRNA and thus MUC2 expression, it has been found that miR-34c could be a regulatory gene of MUC2 [60]. AF147447 was expressed highly when miR-34c was high and vice versa [60]. These results show that lncRNA-AF147447 and miR-34c are positively correlated [60]. Furthermore, MUC2, EGFR, and CD44 are miR-34c targets. In an experiment, it was detected that the expression of EGFR and CD44 is against lncRNA-AF147447. Altogether, these findings determined that lncRNA controls MUC2 expression not only by attaching directly but also via the posttranscriptional pathway, like controlling the miRNA expression [60]. Considering the role of MUC2 in cancer development, it could be a diagnostic biomarker and also a drug aim [60].

Transcriptional factor E2F1 located in the AF147447 transcriptional element attaches to the promoter region of lncRNA and represses their expression [60]. *H. pylori* infection through a transcriptional factor E2F1 decreases lncRNA AF147447 expression [60]. The *H. pylori* infection-related lncRNA AF147447 also functions as a tumor inhibitor through targeting MUC2 and overexpressing miR-34c [3] (Figure 2).

Table 2 shows a list of lncRNAs that are dysregulated in GC cells.

### 7.1. Immunological Procedures

This microorganism stimulates the innate and adaptive immune system; although not destroyed, it causes pathological changes in the gastric mucosa [25]. *H. pylori* stimulates GC cells and epithelial cells in the gastric mucosa to release cytokines such as IL-1*β*, IL-6, IL-8, and tumor necrosis factor- (TNF-) *α*. These cytokines are crucial mediators of gastric pathophysiology and may have important roles in the development of gastric inflammation and GC [4]. *H. pylori* stimulates IL-8 secretion in gastric epithelial cells through the classical activation pathway of NF-*κ*B signaling, which regulates several malignancies in the gastrointestinal tract [4]. It has been determined that *H. pylori* via inducing catalytic activity of the inhibitor of NF-*κ*B (I*κ*B) kinases (IKK*α* and IKK*β*) elevates I*κ*B degradation in GC [4]. It has been shown that *H. pylori* infection inhibits I*κ*B*α* and induces I*κ*B*α* phosphorylation and nuclear p65 expression in SGC-7901 cells, showing that *H. pylori* infection promotes the NF-*κ*B signaling pathway. The activation of NF-*κ*B and the upregulation of IL-8 in GC cells are important mechanisms in *H. pylori*-induced chronic inflammation and gastric carcinogenesis. H19 increases the ability of *H. pylori* to inhibit I*κ*B*α* expression and induces the expression of p-I*κ*B*α* and nuclear p65. Elimination of I*κ*B*α* and increasing of p-I*κ*B*α* and nuclear p65 were done through high expression of H19, abolished by NF-*κ*B inhibitors, BAY11–7082 and pyrrolidine dithiocarbamate (PDTC). Hence, treatment with BAY11–7082 and PDTC reduced proliferation and invasion of *H. pylori*-infected H19 cells. So, in *H. pylori*-infected H19 cells, levels of TNF-*α*, IL-1*β*, IL-6, and IL-8 are increased, but these changes were undone by BAY11–7082 and PDTC. These findings identified that H19 developed proliferation, migration, and invasion of *H. pylori*-infected GC cells through activating the NF-*κ*B signaling pathway. Activation of NF-*κ*B via *H. pylori* in GC cells was mostly by the classical pathway, which depends on *cag*A and its pathogenicity island [4].

The article "Dysregulation of lncRNA in Helicobacter pylori-Infected Gastric Cancer Cells" was published in 2021. Journal: Biomed Res Int.

The cancer-related pathway “PI3K-Akt signaling pathway” is associated with *H. pylori* infection; virulence factors of this bacterium like *cagA* could repress the autophagy through phosphatidylinositol 3′-kinase- (PI3K-) Akt signaling pathway to promote gastric inflammation, subsequently promoting gastric carcinogenesis [58].

In a study, the expression level of cell adhesion molecules like fibronectin 1 (FN1), integrin, CD44, ICAM-1, E-cadherin, N-cadherin, and Vimentin that have previously been confirmed to have a role in invasion and metastasis in various cancers was measured. FN1 was reported to change among them. FN1 is an extracellular matrix glycoprotein that contributes in cell differentiation, growth, and migration. When *FENDRR* was highly expressed, FN1 mRNA was reduced and vice versa [65]. Matrix metalloproteinases (MMPs) are involved in cell invasion and metastasis in human carcinomas [65, 66]. Also indicated was that *FENDRR* potently decreased the activity of MMP2/MMP9 in GC cells, and repression of *FENDRR* leads to the activation of MMP2/MMP9. These findings indicate that FN1 knockdown through downregulation of MMP2 and MMP9 inhibits invasion in gastric carcinoma cells [65].

miRNAs can control the expression of the immune response mediators, and the miRNA expression can be altered by inflammatory mediators [67]. miRNAs contribute significantly in the regulation of inflammatory response related to *H. pylori* infection [15, 68]. The production of IL-6 is decreased through miR-155 and miR-146b in *H. pylori* (cagA+)-induced gastroduodenal ulcers [69]. Inactivation of let-7 miRNAs was found in clinical samples containing *H. pylori*, especially those infected with cagA-positive strains [15, 68]. cagA-positive strains have a role in the inflammatory response, since this virulence factor elevates the production of IL-1*β* and IL-8 and activation of NF-*κ*B, contributes in the process of carcinogenesis, induces growth factors, and inhibits apoptosis. Furthermore, cagA increases oncogenic cells that are important in the pathogenesis of *H. pylori*. In a study, it was determined that *cagA* stimulates miR-223-3p expression by the NF-*κ*B pathway. The oncogenic role of miR-223-3p was confirmed through inhibiting ARID1A (AT-rich interactive domain-containing protein 1A) expression. So these findings show that the NF-*κ*B/miR-223-3p/ARID1A axis may cause the process of *H. pylori*-induced chronic inflammation which leads to gastric cancer and miR-223-3p may apply as a target for the intervention of the malignancy [70]. The VacA factor stimulates a proinflammatory response and helps bacteria to colonize in the gastric mucosa. It has been shown that high expression of VacA results in the production of TNF-*α*, IL-1*β*, nitric oxide, and reactive oxygen species and the activation of NF-*κ*B that are associated with proinflammatory cytokines and apoptosis. VacA through inhibiting phagocytosis and also T cell proliferation enables *H. pylori* to evade the adaptive immune response [67].

The article "Dysregulation of lncRNA in Helicobacter pylori-Infected Gastric Cancer Cells" was published in 2021. Journal: Biomed Res Int.

It has been reported that high expression of miR-21 was related to increased cellular proliferation and antiapoptosis in *H. pylori*-positive gastric tissues; also, miR-146a and miR-155 participated in the weakening of the proinflammatory responses against *H. pylori* [25]. MicroRNA-29c (miR-29c) by targeting integrin subunit beta 1 (ITGB1) has a role in tumor inhibition in GC [24]. In the start of gastric carcinogenesis, the expression of miR-29c is lost and can be used for diagnosis and therapy of GC patients [24]. *H. pylori cag*A induces inactivating of lethal-7 (let-7) expression abnormally, so it leads to renin-angiotensin system (Ras) upregulation and finally GC [24].

## 8. Conclusion and Future Perspectives

In this review, we have brought a subset of inapt lncRNA macromolecules in *H. pylori*-infected gastric mucosa tissues. The studies cleared that lncRNAs are helpful for public health in the area of prevention, diagnosis, and therapy. Many lncRNAs may have crucial roles in the development of cancer. Some of them are involved in the development of *H. pylori*-related diseases. However, there are many issues that remain to be solved. The mechanism of these molecules needs to be understood completely to produce new methods for the therapies of *H. pylori*-related gastric cancer.

There is seldom a study about the ceRNA network related to *H. pylori* infection. Thus, it is expected that the roles of ceRNA regulation in *H. pylori*-infected gastric cancer be investigated. Also, the roles of other lncRNAs should be validated.

The article "Dysregulation of lncRNA in Helicobacter pylori-Infected Gastric Cancer Cells" was published in 2021. Journal: Biomed Res Int.

The significant difference in the results may be attributed to sample size in the study population, genetic background, and genotyping techniques. Follow-up studies are needed to thoroughly understand the value of lncRNA in GC risk and confirm the association between various lncRNAs and GC risk in a large sample size.

In addition, studies should investigate the association between lncRNAs and various virulence factors of *H. pylori* such as cagA, VacA, iceA, sabA, and babA and also survey the relationship between these virulence factors and expression of lncRNAs in various gastrointestinal diseases.

## Figures and Tables

**Figure 1:** lncRNA and related diseases. Expressed lncRNAs are related to various diseases, including infectious diseases, neurological disorders, cardiovascular diseases, and different cancers.

**Figure 2:** *H. pylori* infection through transcriptional factor E2F1 decreases lncRNA AF147447 expression. The *H. pylori* infection-related lncRNA AF147447 functions as a tumor inhibitor through targeting MUC2 and controls MUC2 expression by attaching.

**Table 1:** Subtypes of lncRNA introduced according to the recent studies.

Name	Length (nt)	Function	Example	References
Intergenic	828	Control the expression of both near and remote genes	LINC00152, *H19*, *IPW*, MEG3	[35–37]
Intragenic	—	Attach to promoters and enhancers	RUNXOR	[35, 39]
Enhancer	—	Specific enhancer–promoter looping, gene expression	IG-DMR eRNAs	[35, 56]
Antisense	—	Gene regulation, X-inactivation, imprinting, and epigenetic regulation	*KCNQ1OT1*, *AIRN*, *NESPAS*, *Ube3a-ATS*, ANRIL	[42–44]
sno-lncRNAs	—	Contribute in the pathogenesis of PWS	*—*	[42–44]
circRNAs	Under 100 nt to over 4 kb	Related with disease phenotype	cANRIL	[42–45]
ciRNAs	—	Gene transcription	*—*	[42–45]

lncRNAs: long noncoding RNAs; LINC00152: long intergenic non-protein-coding RNA152; IPW: imprinted gene in the Prader-Willi syndrome region; MEG3: maternally expressed gene 3; RUNXOR: RUNX1 overlapping RNA; IG-DMR: intergenic differentially methylated region; KCNQ1OT1: KCNQ1 opposite strand/antisense transcript 1; AIRN: antisense of insulin-like growth factor-2 receptor RNA noncoding; UBE3A-ATS: UBE3A antisense transcript; ANRIL: antisense noncoding RNA in the INK4 locus.

**Table 2:** Differentially expressed lncRNAs in GC cells.

Upregulated	Downregulated
XIST, H19, LINC00152, THAP9-AS1, HULC, XULC, XLOC-014388, XLOC-004122, LINCO1254, LINCO1287, LINCO1524, U95743.1	FER1L4, CUDR, LSINCT-5, PTENP1, LINC00673, AF147447

## Data Availability

We declare all data are available upon request to the corresponding author.
